# Superficial Retinal Vessel Density and Foveal Avascular Zone in Myopic Anisometropia: An OCTA-Based Study in Young Chinese Children

**DOI:** 10.1155/2022/1229009

**Published:** 2022-07-06

**Authors:** Fen Xiong, Tian Mao, Junchen Wang, Jinglin Yi, Yang Hu, Hongfei Liao

**Affiliations:** ^1^Affiliated Eye Hospital, Nanchang University, Nanchang 330006, China; ^2^West China Medical Center of Sichuan University, Chengdu 610000, China

## Abstract

This retrospective study investigated superficial retinal vessel density (SRVLD) and foveal avascular zone (FAZ) area using optical coherence tomography angiography (OCTA) in children with myopic anisometropia. We included 84 eyes of 42 individuals with myopic anisometropia and no posterior segment abnormalities. All eyes underwent OCTA. Individual SRVLD and FAZ area were measured on OCTA. Using a paired *t*-test, we compared the interocular difference between the fellow eyes for all the measurements. SRVLD was significantly higher in the relatively more myopic eyes than in the fellow eyes in the whole population and in patients with an interocular difference of >1.5 D (*p* = 003 and 0.01, respectively). In patients with an interocular difference of ≤1.5 D in spherical equivalent refraction, only the nasal sector showed higher SRVLD in the less myopic eyes. SRVLD in the whole image and parafoveal sector was significantly lower in the dominant eye (paired *t*-test, *p* = 003 and 0.03, respectively), while other locations showed no difference. The area, perimeter, and circularity index in FAZ parameters showed no difference. SRVLD showed no significant differences between the two types of eyes, with an interocular difference of ≤1.5 D but increased in the relatively more myopic eyes than in the fellow eyes in children with myopic anisometropia, with an interocular difference of >1.5 D. Increasing SRVLD may show a compensatory increase to maintain retinal function and thus maintain normal visual function in the relatively more myopic fellow eyes. As the study to use patients as self-control with OCTA analysis in both eyes, this study provides some reference value for further interpretation of the pathogenesis of anisometropia.

## 1. Introduction

Myopic anisometropia or anisomyopia is commonly detected in school-age children with myopia and progresses with age [1, 2]. It is an unequal refractive state of the eyes, referring to a between-eye difference in myopic spherical equivalent refractive (SER) errors of ≥1.00 D (usually because of an interocular asymmetry in the axial length [AL]), in which the fellow eyes of an individual have grown to two distinctly different endpoints [3]. Severe anisometropia is the causative factor for amblyopia and subnormal binocularity (visual fatigue, diplopia, and declined stereovision) [4].

As a fast, noninvasive technology, OCTA has been widely used in research and clinical diagnosis of retinal microvascular diseases. OCTA can quantitatively and comprehensively analyze the function of ocular blood flow and yield precise details about the structure and microcirculation of the retinal layers for the treatment of retinal vascular images [5]. The retinal capillary network and microcirculation provide the retinal tissue with oxygen and nutrients directly, which could be more likely to induce changes related to myopia. The density of the retinal microvasculature decreased, and longer AL in the eyes with myopia was recorded by several researchers, which may be a potential indication of progressive myopia [6, 7]. Only few studies have focused on retinal biometrics in myopic anisometropia, although many studies have assessed the interocular symmetry of retinal thickness and blood flow in amblyopic anisometropia [8, 9].

There is a need for a study on myopic anisometropia so that it could contribute to potential new insights into the mechanisms of refractive error development. Because these studies compare the less myopic eyes to the relatively more myopic fellow eyes in the same subject, it allows for greater control of confounding variables such as age, gender, genetics, learning ability, and living habits (environment). Therefore, in this study, we aimed to investigate the superficial retinal vessel density (SRVLD) and foveal avascular zone (FAZ) area in children with myopia anisometropia using OCTA and to assess whether ocular dominance may have on the retinal capillary microcirculation.

## 2. Materials and Methods

### 2.1. Participants

Data from subjects who sought vision correction from March 2019 to March 2020 at Nanchang University Affiliated Eye Hospital were reviewed in this current retrospective study. The inclusion criteria are listed in Table 1.

SER was calculated as the addition of the spherical power and half the magnitude of the cylinder power. Aniso-SER was defined as the interocular absolute difference in SER. In this study, we named SER ≥ −0.50 D as nonmyopia.

The study was performed in adherence to the tenets of the Declaration of Helsinki. All parents declared that their children were healthy. All children and their parents were informed about the study procedure, and signed informed consent was obtained from the guardians of all the participants. Ethical approval for the study was obtained from the Nanchang University Clinical Research Centre.

Each enrolled patient underwent complete ophthalmologic examination including monocular best corrected visual acuity testing using a linear logarithm of the minimum angle of resolution (logMAR) charts, intraocular pressure (IOP) measurement using noncontact tonometry equipment (model NT-4000, Nidek Inc., Fremont, CA, USA), slit-lamp examination (Haag-Streit Slit-Lamp, Köniz, Switzerland), and dilated fundus examination with direct ophthalmoscopy, cycloplegic refraction, AL, and anterior chamber depth (ACD) measurement using the IOL Master (Carl Zeiss Meditec Inc., Dublin, CA). Pupillary dilation was induced by the instillation of three drops of 1% cyclopentolate in each eye (Cyclogyl; Alcon, Fort Worth, TX, USA) at 10 min intervals, following which the pupil size and light reflex were examined. Cycloplegia was deemed complete if the pupil had dilated to ≥6 mm and light reflex was absent. An autorefractometer (ARK-700A, Nidek, Japan) was set to generate five valid refraction readings, and the median value recorded by the instrument was used for analysis.

### 2.2. OCTA Scan Protocol and Image Analysis

One expert operator completed all the OCTA examinations with a 3 × 3 mm volume scan pattern centered on the fovea by using Carl Zeiss Cirrus HD-OCT Model 5000. This device used a wavelength of 840 nm. The Zeiss Cirrus HD-OCT Model 5000 with AngioPlex uses a so-called OCT microangiography complex algorithm (OMAG) and an A-scan rate of 68 KHz. OMAG identifies changes in the phase and intensity information of the OCT scans to quantify motion contrast [10]. For eye tracking, the FastTrac technology is implemented and the retina is sampled at a rate of 15 frames per second to minimize motion artifacts. Only areas that may be affected by motion artifacts are rescanned, which decreases the acquisition time. A 3 × 3 pattern with a 245 × 245 resolution was chosen, with a mean distance of 12.2 microns between each scan, and each B-scan was repeated 4 times in the same position. The A-scan depth is 2 mm with an axial resolution of 5 *μ*m and a transverse resolution of 15 *μ*m [10].

Superficial retinal vessel density (SRVLD) was defined as the area occupied by vessel lumens following binary reconstruction of images [11]. Perfusion density (PD) was expressed as the ratio between the measured vessel pixels and the total scan area after subtracting the FAZ area, thus being a dimensionless quantity [12]. The Cirrus HD-OCT review software program automatically calculates the vessel density and PD of the superficial capillary plexus inside these circles and in different sectors (temporal, superior, nasal, and inferior) of the foveal and parafoveal areas (Figure 1). The FAZ area (mm^2^), FAZ perimeter (mm), and circularity index (the ratio between the measured perimeter and the perimeter of a circular area of the same size) were determined automatically using Cirrus HD-OCT review software (Figure 1).

### 2.3. Statistical Analyses

Statistical analyses were conducted using IBM SPSS Statistics, version 23.0 (IBM Co., Armonk, NY, USA). The variables were investigated using visual histograms, probability plots, and the Shapiro-Wilk test to determine whether they were normally distributed. Statistical power analysis was also performed. Descriptive analyses were presented as means and standard deviations (SDs), as the variables were normally distributed. A paired *t*-test was used to compare the interocular difference between the fellow eyes for all the measurements. A *p* value of less than 0.05 indicated statistical significance.

## 3. Results

A total of 84 eyes from 42 patients with myopia anisometropia were enrolled in this study. Twenty-two patients (52.38%) were female. The characteristics of the more and less myopic eyes of the anisometropic subjects are summarized in Table 2 and Figure 2. ACD and AL were significantly shorter in the less myopic eyes (ACD 3.59 ± 0.19 mm and AL 23.82 ± 0.80 mm) than in the relatively more myopic fellow eyes (ACD 3.64 ± 0.18 mm and AL 24.68 ± 0.82 mm, both *p* < 0001). AL/CRC in the less myopic eyes (3.05 ± 0.08) was smaller than that in the relatively more myopic fellow eyes (3.17 ± 0.09), with a significant difference. The CRC and IOP showed no difference between the two groups (*p* = 059 and 0.18, respectively). The clinical parameters in the dominant and nondominant eyes are summarized in Table 3. IOP, SER, ACD, AL, CRC, and AL/CRC showed no significant difference between the two groups (*p* = 024, 0.41, 0.50, 0.49, 0.32, and 0.41, respectively).

### 3.1. Vessel Length Density of the Superficial Plexus

In the entire population and in patients with an interocular difference of >1.5 D, there were no significant differences between the less myopic and the fellow eyes for SRVLD measurement at any of the retinal locations measured (paired *t*-test) except in the foveal sector (*p* = 003 and 0.01, respectively) (Table 2). As for the parafoveal area of the fovea, the nasal sector showed higher SRVLD in the less myopic eyes in patients with an interocular difference of ≤1.5 D in SER (*p* = 004) (Table 2). Furthermore, SRVLD in the relatively more myopic fellow eyes showed a higher score in patients with an interocular difference of more than 1.5 D in SER, but only the inferior sector showed a significance difference (*p* = 004, Figure 2, Table 2). SRVLD values at the whole image and the parafoveal sector were significantly lower in the dominant eye (paired *t*-test, *p* = 003 and 0.03, respectively), while other locations showed no significant difference (Table 3). In addition, neither AL nor AL/CRC had a significant correlation with SRVLD (Table 4).

### 3.2. Perfusion Density

There were no significant differences between the less myopic and the fellow eyes for measures of PD at any of the retinal locations measured (paired *t*-test) (Table 2). The nasal sector showed higher SRVLD in the less myopic eyes in patients with an interocular difference of ≤1.5 D in SER (*p* = 002) (Table 2). In the entire population and in patients with an interocular difference of ≤1.5 D, PD values at the whole image, parafoveal sector, and superior part were significantly lower in the dominant eye (paired *t*-test, *p* = 002, 0.04, and 0.04 vs. 0.01, 0.02, and 0.01, respectively) (Table 3). Furthermore, PD values at the foveal part were significantly lower in the dominant eye in patients with an interocular difference of ≤1.5 D (*p* = 004).

### 3.3. FAZ Parameters

The area, perimeter, and circularity index in the FAZ parameters showed no significant difference in all the groups (Tables 2 and 3).

## 4. Discussion

Our result could invalidate the hypothesis that patients with higher degree of myopia suffer less SRVLD as it indicates that higher degree of myopia suffered more SRVLD when the interocular difference > 1.5 D. Furthermore, the nondominant eye had a higher SRVLD when the interocular difference ≤ 1.5 D.

Some previous studies showed the myopic eyes exhibited a larger area of foveal avascular zone than the control groups [6, 13] which is in contrast with our result. The FAZ parameters showed no significant difference in all the groups. The difference in the results between previous studies and the present study could be explained by the different study population.

Regarding the SRVLD at the whole image, foveal sector, and parafoveal sector, we found no significant differences between the two eyes with an interocular difference of ≤1.5 D in SER. However, when we focused on the whole patients and patients with an interocular difference of >1.5 D in SER, we found a significantly higher value in the relatively more myopic eyes than in the fellow eyes (*p* = 001 and 0.03, respectively). As for the parafoveal area of the fovea, all the sectors showed a higher SRVLD in the less myopic eyes except for the temporal sector in patients with an interocular difference of ≤1.5 D in SER. Furthermore, the relatively more myopic fellow eyes showed higher SRVLD in patients with an interocular difference of >1.5 D in SER. Li et al. indicated that the longer axial eyes had higher superficial macular vessel density and lower radial peripapillary capillary density than did the contralateral eyes in patients with myopic anisometropia [14]. This research showed the same result with us in the patients with an interocular difference of >1.5 D in SER or the whole group. Most notably, several studies have shown a significantly higher value of SRVLD in emmetropia subjects than in myopic subjects [7, 15, 16]. Furthermore, the decrease in SRVLD was significantly correlated with AL in high myopia [7, 17, 18]. We believe that the choroidal thickness is thinner in the more myopic eyes, and the vascular density of the choriocapillaris is reduced in the more myopic eyes of children with anisometropia, which also may lead to a thinner retina [19–21]. The findings reported in all the studies were consistent with our result in patients with an interocular difference of ≤1.5 D in SER but were in contrast with our result in patients with an interocular difference of >1.5 D in SER.

We considered a different study population, and several anatomical changes may have led to this discrepancy. Our study population included two eyes from one patient, which indicates paired samples, while the other studies included independent samples.

In other studies, while macular flow densities were found to be decreased in pathological myopia compared with high myopia and emmetropia, there was no significant decrease in retinal flow density in the macular area in the high myopic eyes compared with that in the emmetropic eyes [7]. Furthermore, the SRVLD showed a positive correlation with retinal thickness at all macular locations, especially in the foveal region [22] and the ganglion cell layer-inner plexiform layer complex [23]. Thus, we focused on the macular thickness in myopic anisometropia. The macular thickness was found to be significantly increased in the relatively more myopic eyes versus the fellow eyes in the lower levels of myopic anisometropia (1.5 D to 3.00 D), and there were no obvious structural differences between the two eyes in regard to the macula or the paramacular regions [24]. Additionally, the minimum and average foveal thicknesses were found to be significantly thicker in the highly myopic eyes than in the fellow eyes when retinal characteristics were examined in severe myopic anisometropia (approximately 10.0 D) [25]. Findings from these clinical studies are consistent with our result where the SRVLD at the foveal sector showed a higher value in the relatively more myopic eyes than in the fellow eyes. The vascular plexus in the superficial macular area mainly supplies nutrients to the retinal nerve fiber layer, ganglion cell layer, and inner plexiform layer [26]. An increased SRVLD may be a compensatory to maintain the retinal function and thus retain normal visual function in the relatively more myopic fellow eyes. Therefore, it seems that an increased SRVLD may initially occur in the inferior and the foveal sector when the interocular difference becomes bigger.

We found an interesting phenomenon in terms of ocular dominance; the SRVLD values at the whole image and the parafoveal sector were significantly higher in the nondominant eye, especially in patients with an interocular difference of ≤1.5 D in SER. The dominant eye has greater degree of myopia than the nondominant eye in some subjects with anisometropic myopia. When anisometropia exceeded 1.75 D, the difference was more evident in 90% of subjects [27, 28]. It is well known that retinal and choroidal thickness is thinner in the more myopic eyes. The vascular density of the choriocapillaris is reduced in the more myopic eyes of children with anisometropia [19, 21, 29]. Additionally, we speculate that this may be due to the lag of accommodation. The dominant eye has a greater degree of myopia [27, 28] and thus gains a hyperopic defocus due to the greater lag of accommodation [30]. As a consequence, choroidal thickness decreases [19, 21, 31, 32], which may lead to a thinner retina and a decreased SRVLD [33]. Therefore, we have considered that a greater degree of myopia (a longer axial length) in the dominant eye may lead to a thinner retina and a decreased SRVLD [33] in all the patients with myopic anisometropia, although the difference was not statistically significant in the patients with an interocular difference of >1.5 D. Studies of over 10,000 patients also found that in myopic anisometropia, the dominant eye is typically the eye with the lower refractive error [34, 35]. Thus, differences in subject ethnicity and age may account for some of the discrepancies observed in the findings between the studies.

Our analysis has some drawbacks. To begin with, the participants in our study's stage of myopia and anisometropia were clustered in a small area, and the age of the patients was limited in teenager classes. Therefore, a wider selection of participants can be obtained in the future analysis to obtain a more compelling and detailed conclusion.

Our study has a few limitations. Our research is limited by our OCTA instrument; it only allowed us to measure the superficial retinal vascular plexus. We consider that deeper retinal plexuses would be presented the similar outcome, or even more significant influence, which would imply the metabolism to the retina is more widespread than implied by the current findings. Another limitation of our study is the relatively few subjects in this study.

## 5. Conclusions

Our results provide evidence that patients with higher degree of myopia have a lower SRVLD. SRVLD showed no significant differences between the two eyes in children with an interocular difference of ≤1.5 D but increased in the relatively more myopic eyes than in the fellow eyes in myopic anisometropia children with an interocular difference of >1.5 D. Increasing SRVLD may show a compensatory increase to maintain retinal function and thus retain normal visual function in the relatively more myopic fellow eyes. We also found the SRVLD values were significantly lower in the dominant eye, especially in patients with an interocular difference of ≤1.5 D in SER. We have considered that lag of accommodation and long axial length have attributed to it. As a study to use patients as self-control with OCTA analysis in both eyes, this study provides some reference value for further interpretation of the pathogenesis of anisometropia.

## Figures and Tables

**Figure 1:** (a) Retinal segmentation at optical coherence tomography (OCT) angiography. (b) The superficial retinal vessel density. (c) The superficial retinal perfusion density. (d) The colored lines in horizontal OCT B-scans show segmentation lines that define the different depth in the retinal tissue of the superficial capillary plexus. (e) Graphic representation of retinal area evaluated at OCT angiography. The software selected the 3 × 3 mm image with 2 rings of 3.0 and 1.0 mm diameter centered on the fovea. The vessel density was calculated for the whole 3 mm circle area centered on the fovea (whole image) (1E), for the area inside the central 1 mm circle (foveal sector) (2E), for the area between the outer 3 mm circle and the inner 1 mm circle (parafoveal sector) (3E).

**Figure 2:** Vessel length density of the superficial plexus in different sectors. Solid lines represent the patients with interocular difference ≤ 1.5 D in SER. Dotted lines represent the patients with interocular difference > 1.5 D in SER.

**Table 1:** Inclusion criteria.

Age	6-16 years
Refraction	−6.00 D < SER < −0.50 D in one eye
	Aniso-SER no less than 1.00 D
	Astigmatism no more than 3.00 D
BCVA	Equal to or better than 0.1 (logMAR) in each eye
Ocular health	Had no other ocular diseases aside from refractive error
	No amblyopia or strabismus
	No pathological myopia
Others	No previous history of ocular disease or surgery
	OCTA images with SSI > 70 and QI > 7

SER: spherical equivalent refraction; OCTA: optical coherence tomography angiography; SSI: signal strength index; QI: quality index.

**Table 2:** The clinical parameters between the different myopia groups.

Variables	Less myopic eyes	The fellow relatively more myopic eyes	*p*	Less myopic eyes	The fellow relatively more myopic eyes	*p*	Less myopic eyes	The fellow relatively more myopic eyes	*p*
	All patients			The patients with interocular difference ≤ 1.5 D in SER			The patients with inter-ocular difference > 1.5 D in SER		
Number of eyes	47.00	47.00		20.00	20.00		27.00	27.00	
Age (year)	13.62 ± 3.95			14.04 ± 3.78			13.58 ± 3.19		
IOP (mmHg)	16.00 ± 3.20	16.35 ± 3.07	0.59	16.47 ± 3.53	16.42 ± 3.49	0.91	15.57 ± 3.03	16.29 ± 3.02	0.07
SER (D)	−0.51 ± 1.02	−2.49 ± 1.29	<0.001	−0.50 ± 0.22	−1.65 ± 1.19	<0.001	−0.52 ± 0.42	−3.22 ± 1.28	<0.001
ACD (mm)	3.59 ± 0.19	3.64 ± 0.18	<0.001	3.58 ± 0.16	3.61 ± 0.17	<0.001	3.61 ± 0.27	3.66 ± 0.18	<0.001
AL (mm)	23.82 ± 0.80	24.68 ± 0.82	<0.001	22.78 ± 0.70	24.26 ± 0.82	<0.001	23.81 ± 0.6	24.95 ± 0.67	<0.001
CRC (mm)	7.79 ± 0.26	7.78 ± 0.25	0.18	7.75 ± 0.27	7.73 ± 0.24	0.19	7.82 ± 0.24	7.83 ± 0.15	0.15
AL/CRC	3.05 ± 0.08	3.17 ± 0.09	<0.001	3.07 ± 0.08	3.14 ± 0.09	<0.001	3.05 ± 0.11	3.2 ± 0.11	<0.001

Vessel length density (mm^−1^)									
Whole image	20.28 ± 1.34	20.48 ± 1.22	0.37	20.42 ± 1.16	20.18 ± 1.30	0.46	20.16 ± 1.49	20.72 ± 1.13	0.08
Foveal sector	9.93 ± 2.50	10.57 ± 3.04	**0.03**	9.83 ± 2.84	10.06 ± 3.63	0.60	10.01 ± 2.26	10.99 ± 2.5	**0.01**
Parafoveal sector	21.61 ± 1.36	21.74 ± 1.10	0.58	21.79 ± 1.20	21.46 ± 1.11	0.30	21.46 ± 1.49	21.96 ± 1.05	0.12
Superior	21.41 ± 1.68	21.51 ± 1.42	0.76	21.57 ± 1.81	21.18 ± 1.22	0.41	21.29 ± 1.6	21.77 ± 1.55	0.22
Inferior	21.72 ± 1.49	22.03 ± 0.98	0.17	21.94 ± 1.12	21.76 ± 0.98	0.52	21.55 ± 1.74	22.25 ± 0.95	**0.04**
Nasal	22.21 ± 1.40	21.78 ± 1.47	0.18	22.24 ± 1.41	21.15 ± 1.54	**0.04**	22.18 ± 1.43	22.3 ± 1.2	0.74
Temporal	21.07 ± 1.96	21.61 ± 1.85	0.27	21.43 ± 1.69	21.74 ± 1.78	0.63	20.79 ± 2.14	21.5 ± 1.95	0.32

Perfusion density ([white pixels/(white + black pixels)] × 100)									
Whole image	0.36 ± 0.02	0.36 ± 0.02	0.99	0.36 ± 0.02	0.36 ± 0.02	0.53	0.36 ± 0.03	0.37 ± 0.02	0.34
Foveal sector	0.17 ± 0.04	0.18 ± 0.05	0.08	0.16 ± 0.05	0.17 ± 0.06	0.52	0.38 ± 0.03	0.38 ± 0.03	0.05
Parafoveal sector	0.38 ± 0.02	0.38 ± 0.02	0.75	0.39 ± 0.02	0.38 ± 0.02	0.32	0.38 ± 0.03	0.39 ± 0.01	0.54
Superior	0.38 ± 0.03	0.38 ± 0.03	0.51	0.38 ± 0.03	0.38 ± 0.03	0.65	0.4 ± 0.03	0.4 ± 0.03	0.23
Inferior	0.39 ± 0.02	0.39 ± 0.02	0.61	0.39 ± 0.02	0.39 ± 0.02	0.62	0.37 ± 0.04	0.38 ± 0.04	0.28
Nasal	0.40 ± 0.03	0.38 ± 0.03	0.06	0.4 ± 0.03	0.37 ± 0.03	**0.02**	0.17 ± 0.04	0.19 ± 0.04	0.74
Temporal	0.37 ± 0.04	0.38 ± 0.04	0.33	0.38 ± 0.04	0.39 ± 0.04	0.41	0.38 ± 0.03	0.39 ± 0.01	0.55

FAZ parameters									
Area (mm^2^)	0.29 ± 0.10	0.27 ± 0.11	0.06	0.31 ± 0.13	0.3 ± 0.14	0.29	0.27 ± 0.06	0.24 ± 0.08	0.12
Perimeter (mm)	2.24 ± 0.38	2.14 ± 0.51	0.17	2.04 ± 0.58	2.11 ± 0.50	0.11	2.46 ± 0.14	2.17 ± 0.21	0.22
Circularity index	0.70 ± 0.09	0.71 ± 0.09	0.61	0.72 ± 0.04	0.75 ± 0.07	0.72	0.68 ± 0.12	0.68 ± 0.11	0.60

ACD: anterior chamber depth; CRC: corneal radius of curvature; AL: axial length. ^∗^Paired *t*-test.

**Table 3:** The clinical parameters in the dominant and nondominant eye.

Variables	Dominant eye	Nondominant eye	*p* ^∗^	Dominant eye	Nondominant eye	*p* ^∗^	Dominant eye	Nondominant eye	*p* ^∗^
	All patients			The patients with interocular difference ≤ 1.5 D in SER			The patients with interocular difference > 1.5 D in SER		
Number of eyes	47.00	47.00		20.00	20.00		27.00	27.00	
Age (year)	13.62 ± 3.95			14.12 ± 2.38			13.36 ± 3.39		
IOP (mmHg)	15.96 ± 2.10	16.09 ± 2.07	0.24	16.47 ± 3.41	16.42 ± 3.61	0.91	16.3 ± 3.47	15.65 ± 2.68	0.11
SER (D)	−1.33 ± 1.62	−1.62 ± 1.44	0.41	−1.06 ± 0.7	−1.16 ± 0.75	0.69	−1.52 ± 2.16	−2.08 ± 1.78	0.38
ACD (mm)	3.62 ± 0.19	3.61 ± 0.18	0.50	3.61 ± 0.19	3.57 ± 0.21	0.15	3.62 ± 0.2	3.64 ± 0.18	0.34
AL (mm)	24.17 ± 0.83	24.27 ± 0.97	0.49	24.07 ± 0.6	24 ± 0.76	0.58	24.22 ± 0.99	24.53 ± 1.11	0.24
CRC (mm)	7.79 ± 0.26	7.78 ± 0.25	0.32	7.69 ± 0.27	7.71 ± 0.24	0.89	7.84 ± 0.24	7.79 ± 0.15	0.23
AL/CRC	3.11 ± 0.10	3.12 ± 0.10	0.41	3.11 ± 0.06	3.1 ± 0.06	0.97	3.11 ± 0.13	3.15 ± 0.13	0.28

Vessel length density (mm^−1^)									
Whole image	20.15 ± 1.39	20.64 ± 1.16	**0.03**	19.94 ± 1.19	20.67 ± 1.18	**0.01**	20.28 ± 1.58	20.57 ± 1.19	0.42
Foveal sector	10.13 ± 2.75	10.59 ± 2.75	0.12	9.54 ± 3.08	10.35 ± 3.38	0.05	10.52 ± 2.42	10.68 ± 2.14	0.72
Parafoveal sector	21.43 ± 1.31	21.92 ± 1.14	**0.03**	21.26 ± 1.08	21.98 ± 1.14	**0.02**	21.54 ± 1.52	21.84 ± 1.2	0.40
Superior	21.14 ± 1.65	21.74 ± 1.43	0.05	20.79 ± 1.71	21.95 ± 1.11	**0.01**	21.41 ± 1.63	21.52 ± 1.69	0.80
Inferior	21.73 ± 1.38	22.09 ± 1.13	0.12	21.74 ± 0.79	21.96 ± 1.25	0.41	21.69 ± 1.79	22.16 ± 1.04	0.23
Nasal	21.84 ± 1.39	22.11 ± 1.52	0.39	21.71 ± 1.2	21.68 ± 1.89	0.96	21.94 ± 1.6	22.47 ± 1.06	0.17
Temporal	20.97 ± 1.88	21.72 ± 1.94	0.13	20.82 ± 1.68	22.35 ± 1.41	**0.01**	21.04 ± 2.11	21.19 ± 2.25	0.85

Perfusion density ([white pixels/(white + black pixels)] × 100)									
Whole image	0.36 ± 0.02	0.37 ± 0.02	**0.02**	0.35 ± 0.02	0.37 ± 0.02	**0.01**	0.36 ± 0.03	0.36 ± 0.02	0.40
Foveal sector	0.16 ± 0.05	0.18 ± 0.05	0.11	0.16 ± 0.05	0.17 ± 0.06	**0.04**	0.18 ± 0.04	0.18 ± 0.04	0.80
Parafoveal sector	0.38 ± 0.02	0.39 ± 0.02	**0.04**	0.38 ± 0.02	0.39 ± 0.02	**0.02**	0.38 ± 0.03	0.39 ± 0.02	0.50
Superior	0.37 ± 0.03	0.39 ± 0.03	**0.04**	0.37 ± 0.03	0.39 ± 0.02	**0.01**	0.38 ± 0.03	0.38 ± 0.03	0.70
Inferior	0.38 ± 0.02	0.39 ± 0.02	0.17	0.38 ± 0.01	0.39 ± 0.02	0.44	0.38 ± 0.03	0.39 ± 0.01	0.35
Nasal	0.39 ± 0.03	0.39 ± 0.04	0.54	0.39 ± 0.03	0.38 ± 0.04	0.75	0.39 ± 0.03	0.4 ± 0.03	0.23
Temporal	0.37 ± 0.04	0.39 ± 0.04	0.18	0.37 ± 0.04	0.4 ± 0.03	0.02	0.37 ± 0.04	0.37 ± 0.05	0.99

FAZ parameters									
Area (mm^2^)	0.28 ± 0.10	0.27 ± 0.12	0.51	0.3 ± 0.13	0.31 ± 0.14	0.56	0.27 ± 0.06	0.25 ± 0.09	0.36
Perimeter (mm)	2.22 ± 0.35	2.16 ± 0.53	0.42	2.28 ± 0.41	2.3 ± 0.5	0.70	2.18 ± 0.31	2.04 ± 0.55	0.35
Circularity index	0.71 ± 0.08	0.70 ± 0.10	0.84	0.71 ± 0.08	0.7 ± 0.07	0.82	0.7 ± 0.09	0.7 ± 0.12	0.89

CRC: corneal radius of curvature; AL: axial length. ^∗^Paired *t*-test.

**Table 4:** The correlation of SRVLD with clinical parameters.

			Vessel length density							Perfusion density							
			Superior	Inferior	Nasal	Temporal	Foveal quadrant	Parafoveal quadrant	Whole image	Superior	Inferior	Nasal	Temporal	Foveal quadrant	Parafoveal quadrant	Whole image	FAZ area
AL	Less myopic eyes	*r* ^∗^	0.07	-0.02	0.18	-0.09	0.07	0.05	0.07	-0.01	-0.09	0.14	-0.19	0.23	-0.02	0.00	-.347^∗^
		*p* ^╁^	0.67	0.90	0.25	0.58	0.65	0.74	0.67	0.94	0.60	0.38	0.25	0.15	0.88	0.99	**0.03**
	The more myopic eyes	*r* ^∗^	0.30	0.25	0.18	0.19	0.18	0.27	0.27	0.25	0.27	0.08	0.08	0.17	0.25	0.19	-0.08
		*p* ^╁^	0.06	0.12	0.26	0.24	0.28	0.09	0.09	0.12	0.10	0.60	0.63	0.30	0.12	0.23	0.64
	Dominant eye	*r* ^∗^	0.12	0.10	-0.04	-0.04	0.19	0.03	0.07	0.11	0.05	-0.13	-0.17	0.15	-0.08	-0.05	-0.29
		*p* ^╁^	0.46	0.55	0.80	0.79	0.24	0.84	0.65	0.49	0.76	0.43	0.28	0.36	0.64	0.78	0.07
	Nondominant eye	*r* ^∗^	0.19	0.26	0.19	0.23	0.25	0.26	0.30	0.11	0.21	0.07	0.13	0.24	0.19	0.19	-0.15
		*p* ^╁^	0.25	0.12	0.25	0.16	0.13	0.11	0.06	0.49	0.21	0.69	0.43	0.14	0.24	0.24	0.35

AL/CRC	Less myopic eyes	*r* ^∗^	-0.03	-0.11	-0.10	0.07	-0.10	-0.05		-0.02	-0.17	-0.12	0.10	0.00	-0.06	-0.05	-0.10
		*p* ^╁^	0.85	0.48	0.54	0.66	0.52	0.75	0.68	0.88	0.29	0.47	0.54	0.99	0.71	0.78	0.55
	The more myopic eyes	*r* ^∗^	-0.07	0.18	0.24	-0.19	-0.04	0.03	0.03	-0.10	0.16	0.23	-0.29	-0.06	0.00	-0.04	0.04
		*p* ^╁^	0.68	0.28	0.14	0.25	0.82	0.83	0.88	0.53	0.31	0.15	0.07	0.72	0.99	0.80	0.80
	Dominant eye	*r* ^∗^	0.04	0.23	0.03	0.12	0.12	0.12	0.13	0.06	0.14	-0.08	0.05	0.08	0.04	0.05	-0.02
		*p* ^╁^	0.81	0.15	0.87	0.46	0.47	0.45	0.43	0.73	0.38	0.62	0.74	0.63	0.82	0.74	0.90
	Nondominant eye	*r* ^∗^	-0.15	-0.08	-0.04	-0.11	-0.07	-0.12	-0.12	-0.16	-0.12	-0.05	-0.12	-0.06	-0.15	-0.16	-0.11
		*p* ^╁^	0.36	0.63	0.82	0.49	0.68	0.45	0.47	0.33	0.47	0.75	0.48	0.70	0.36	0.32	0.50

^∗^Pearson product-moment correlation coefficient. ^╁^Level of statistical significance.

## Data Availability

The data used to support the findings of this study are available from the corresponding authors upon request.
